The article "Indirect Recruitment of a CD40 Signaling Pathway in Dendritic Cells by B7-DC Cross-Linking Antibody Modulates T Cell Functions" was retracted in 2010. Reasons: an official misconduct investigation; misconduct by an author; results that could not be reproduced; concerns about the data.

# Indirect Recruitment of a CD40 Signaling Pathway in Dendritic Cells by B7-DC Cross-Linking Antibody Modulates T Cell Functions

**DOI:** 10.1371/journal.pone.0005373

**Published:** 2009-04-28

**Authors:** Suresh Radhakrishnan, Rosalyn Cabrera, Kristina M. Bruns, Virginia P. Van Keulen, Michael J. Hansen, Sara J. Felts, Larry R. Pease

**Affiliations:** Department of Immunology, College of Medicine, Mayo Clinic, Rochester, Minnesota, United States of America; New York University School of Medicine, United States of America

## Abstract

The human IgM B7-DC XAb protects mice from tumors in both therapeutic and prophylactic settings. Its mechanism of action is mediated by its binding to B7-DC/PD-L2 molecules on the surface of dendritic cells (DCs) to induce a multimolecular cap and subsequent activation of signaling cascades that determine a unique combination of DC phenotypes. One such phenotype, the B7-DC XAb-induced antigen accumulation in mTLR-matured DCs, has been linked to signaling through TREM-2, but the signals required for other DC phenotypes critical for the therapeutic effects in animal models remain unclear. Here, FRET and co-immunoprecipitation studies show that CD40 is recruited to the multi-molecular complex by B7-DC XAb. Signals emanating from CD40 are important, as CD40^−/−^ DCs treated with B7-DC XAb (DC^XAb^) activated DAP12, but failed to activate NFκB, and were not protected from cell death upon cytokine withdrawal or treatment with Vitamin D_3_. CD40^−/−^ DC^XAb^ also failed to secrete IL-6 and were unable to support the conversion of T regulatory cells into IL-17+ effector T cells in vitro. Importantly, the expression of CD40 was required for the overall ability of B7-DC XAb to induce anti-tumor CTL, to provide protection from a number of tumor types, and for DC^XAb^ to be effective anti-tumor vaccines in vivo. These results indicate that B7-DC XAb modulation of DC phenotypes is through its ability to indirectly recruit common signaling molecules and elements of their endogenous signaling pathways through targeted binding to a cell-specific surface determinant.

## Introduction

Generation of a vigorous T cell response is dependent on the activation of the T cells by professional antigen presenting cells and requires stable pMHC∶TCR interaction (signal 1), co-stimulation through CD28 and other membrane molecules (signal 2), and secretion of T cell growth factors (signal 3). B7-DC XAb is an IgM antibody from the serum of a patient with Waldenstrom's macroglobulinemia that binds to the surface of mouse and human DCs [1]. This binding leads to activation of the DCs and an augmentation of a number of phenotypic functions that are distinct from those elicited in DCs activated by TLR ligands or CD40L [2]. The pentameric structure of the IgM antibody is mandatory for the antibody to execute its effect on DCs. Monomers fail to bind and activate the DC and can prevent DC binding by the pentamer [1]. A candidate gene approach revealed that antibody binding is dependent on the expression of the co-stimulatory molecule B7-DC/ PD-L2 [1]. Therefore, we refer to this antibody as B7-DC cross-linking antibody (B7-DC XAb). Importantly, B7-DC XAb also activates human DC [3] and has actions in several experimental models of cancer in which results from the use of TLR ligands or TNF family members have been less impressive [4], [5].

The article "Indirect Recruitment of a CD40 Signaling Pathway in Dendritic Cells by B7-DC Cross-Linking Antibody Modulates T Cell Functions" was retracted in 2010. Reasons: an official misconduct investigation; misconduct by an author; results that could not be reproduced; concerns about the data.

The B7-DC molecule has a short cytoplasmic tail (5 amino acids), does not have charged amino acids, and by itself cannot convey signals from the membrane to the cytoplasm. We have recently shown that treatment of DCs with B7-DC XAb (DC^XAb^) induces multiple membrane proteins to become organized into a cell surface cap [3]. These molecules include B7-1 (CD80), B7-2 (CD86), class-II, TREM-2 and CD11c. Stimulation of antigen accumulation by DC^XAb^ requires TREM-2 and is mediated by the activation of DAP12 and Syk. TREM-2 is also required for B7-DC XAb-mediated tumor protection in mice. However, in subsequent experiments, we found that TREM-2 was dispensable for the activation of an NFκB pathway necessary for DC treated with B7-DC XAb to remain viable under stress [6]. CD40 activation has been shown to increase the viability of a number of cell types including dendritic cells, to activate NFκB, and to increase secretion of a number of cytokines such as IL-1, IL-6 and TNFα [7]–[9]. CD40 activation mechanisms can also lead to tumor immunity [10]–[12]. Thus, we hypothesized that CD40 may play a role in some of the phenotype responses observed in DC^XAb^.

In this report we show that CD40 is indeed present in a B7-DC XAb-induced cell surface complex and is required for activation of NFκB, protection of DC^XAb^ from cell death signals, and for the secretion of IL-6. CD40 expression is also required for DC^XAb^ to reprogram T regulatory cells to IL-17+ effectors, an outcome of B7-DC XAb shown previously to break tolerance in an antigen-specific manner [5]. Finally, presence of CD40 on the DCs in vitro and in vivo is required for the generation of tumor-specific cytolytic effector cells and to protect mice from tumors. Thus B7-DC XAb modulation of DC phenotypes is through its ability to bind a cell-specific molecule to simultaneously recruit and activate multiple signaling cascades in a combinatorial manner to directly regulate DC responses and indirectly regulate T cell functions.

The article "Indirect Recruitment of a CD40 Signaling Pathway in Dendritic Cells by B7-DC Cross-Linking Antibody Modulates T Cell Functions" was retracted in 2010. Reasons: an official misconduct investigation; misconduct by an author; results that could not be reproduced; concerns about the data.

## Results

### B7-DC XAb induces CD40 recruitment into the multi-molecular cap on DCs

Previous dissection of the mechanism of the B7-DC XAb action showed that its binding to DC caused a reorganization of cell surface molecules (class II, CD80, CD86) into a cap-like cluster that also contained the signaling molecule TREM-2 [3]. While DCs from TREM-2 knockout mice were not able to accumulate antigen in response to B7-DC XAb, they were still able to activate NFκB, a mediator of DC viability following B7-DC crosslinking. Since CD40 is a known activator of NFκB, we used FRET analysis to determine whether CD40 was among the cell surface molecules recruited into the B7-DC XAb-induced cap on DC. A FRET signal between the PE-labeled anti-CD40 and APC labeled anti-Class II was detected as early as 5 minutes in DCs stimulated with B7-DC XAb (Fig. 1A, unfilled histograms). Thus, B7-DC XAb cross-linked CD40 to a previously identified constituent of the cell surface cap. The signal was maintained for as long as 30 minutes, but no FRET signal was detected upon stimulation with control antibody (filled histograms). To directly demonstrate that CD40 molecules were present in a multi-molecular complex, we performed Western blots on MHC class II immunoprecipitates. CD40 was detected in MHC class II complexes isolated from the DCs stimulated with B7-DC XAb but not from DCs stimulated with control antibody (Fig. 1B). Taken together, these data suggest that CD40 is recruited into the multimolecular cap that forms on DCs upon treatment with B7-DC XAb.

**Figure 1:** CD40 is rapidly recruited into complexes containing MHC MHC class II on dendritic cells treated with B7-DC XAb. (A) DCs were pre-stained with APC-labeled antibody against MHC class II and PE-labeled antibody against CD40 for 15 min. An aliquot of cells was analyzed by flow cytometry (0 min time point). The remaining cells were then treated with 10 µg/ml IgM control antibody (filled histograms) or B7-DC XAb (open histograms). Cells were sampled at the indicated time points and analyzed for a FRET (FL3 channel). (B) Lysates were prepared from untreated DC (0′) or DC treated with control antibody or B7-DC XAb for the indicated times and subjected to immunoprecipitation using an antibody against MHC class II. The resultant complexes were resolved by SDS-PAGE, transferred to PVDF membrane, and probed for CD40. IgH serves as a loading control. The results shown are representative of 2 experiments.

### CD40 is required for NFκB activation in DC treated with B7-DC XAb

Activation of CD40 culminates in stimulation of NFκB in multiple cell types [8], [13], [14]. Since CD40 was found to complex with class II, we asked whether CD40 mediated NFκB activation in DC^XAb^. Bone marrow derived DCs from wild type, CD40^−/−^, or TREM2^−/−^ mice were stimulated with control antibody or B7-DC XAb for 15 minutes. In addition, parallel CD40^−/−^ DC were stimulated with anti-CD40 or the TLR4 agonist, LPS. Cells were permeabilized and stained with an antibody that recognizes only the activated NFκB complex [6] and visualized by confocal microscopy. Abundant nuclear fluorescence (FITC-anti-p65 alone, upper left panels; merged with DAPI, lower panels) shows that NFκB was activated in wild type and TREM2^−/−^ DCs stimulated with B7-DC XAb but not in CD40^−/−^ (KO) DC stimulated with B7-DC XAb, or anti-CD40 antibody (Fig. 2A). However, CD40^−/−^ DC still activated NFκB when stimulated through TLR4. Control antibody treatment failed to activate NFκB in all groups of DCs. The CD40^−/−^ DCs activated DAP12 and Syk kinase upon B7-DC crosslinking (Fig. 2B), underscoring these cells were only non-responsive to CD40-dependent signals.

The article "Indirect Recruitment of a CD40 Signaling Pathway in Dendritic Cells by B7-DC Cross-Linking Antibody Modulates T Cell Functions" was retracted in 2010. Reasons: an official misconduct investigation; misconduct by an author; results that could not be reproduced; concerns about the data.

**Figure 2:** DCs require CD40 for B7-DC XAb mediated NFκB activation and protection from cell death. (A) NFκB activation in wild type (WT), CD40^−/−^ or TREM2^−/−^ (KO) DC was determined after 15 min stimulation with control antibody, B7-DC XAb, anti-CD40, or LPS (TLR4 ligand). Cells were fixed, stained and imaged using a confocal microscope. Upper left panels show FITC-anti-p65 staining, upper right panels show DAPI staining of nuclei, lower panels show merged images of the upper panels. (B) Wild-type or CD40^−/−^ (KO) DC were treated with control antibody or B7-DC XAb for 5 min. DAP12- (left) or Syk- (middle) specific immunoprecipitates or whole cell lysate for ERK (right) were resolved and blotted using a phosphotyrosine-specific antibody. IgH or total ERK serves as a loading control. (C) Cell death was induced in wild type (filled bars) or CD40^−/−^ (open bars) DC by treatment with vitamin D_3_. All cultures were subsequently incubated with Alamar Blue Dye. Cell viability was measured using a fluorescence plate reader after 24 hours and is expressed as relative fluorescence units (RFU). (D) Similar to (C) except cell death was induced by cytokine withdrawal. Wild type (filled bars) or CD40^−/−^ (open bars) DC were cultured in the presence or absence of GM-CSF and IL-4 (+ or − Cytokine) for 24 h in the presence of 10 µg/ml control antibody, B7-DC XAb, anti-MHC class II IgM antibody 25-9-3, or the combination of 1 µg/ml B7-DC XAb and 0.1 µg/ml RANKL as indicated. The results shown are representative of 2 experiments.

### CD40 is important in promotion of B7-DC cross-linking Ab-induced DC survival under adverse conditions

CD40-CD40L interaction has been shown to promote survival of a number of cell types [15], [16]. Since CD40 was shown to be present in the cell surface complex that forms after cross-linking B7-DC on DCs, we tested whether CD40 was required for the enhanced survival previously observed in DC^XAb^ [6]. Bone marrow derived DCs from wild type or CD40^−/−^ mice were matured with CpG then treated with the cell death inducer Vitamin D_3_ [17]. Cells were then mixed with Alamar Blue dye to determine viability (expressed as mean relative fluorescence). Wild type DCs that received B7-DC XAb remained viable in the presence of Vitamin D_3_ while control antibody failed to protect wildtype DC (Fig. 2C). The effect of B7-DC XAb was dependent on presence of CD40, as DCs that lacked CD40 were not protected from this cell death pathway (Fig. 2C). Wild type or CD40^−/−^ DC were also tested for B7-DC XAb-induced survival when deprived of GM-CSF/IL-4 cytokines for 24 hours. Only wild type DCs treated with B7-DC cross-linking Ab were able to survive cytokine withdrawal, and B7-DC XAb treatment was unable to promote cell survival in CD40^−/−^ DCs. However, CD40^−/−^ DC were still protected cells from cytokine withdrawal if stimulated with RANK ligand, another known activator of NFκB and downstream pro-survival signals (Fig. 2D). CD40 ligation has been demonstrated to activate ERK, and activation of ERK promotes cell survival. Therefore, we tested the requirement for CD40 in ERK activation in response to B7-DC XAb. Wild-type DCs, but not CD40−/− DCs, exhibited ERK activation in response to B7-DC XAb cross-linking, (Figure 2B). Both groups of DCs activated ERK in response to TLR4 ligation. These findings demonstrate that CD40 is an essential upstream mediator of ERK and NFκB activation in DC treated with B7-DC XAb and link CD40 to the enhanced survival phenotype observed in DC^XAb^. Moreover, this pathway is distinct from the TREM2 pathway used by DC^XAb^ to accumulate antigen.

The article "Indirect Recruitment of a CD40 Signaling Pathway in Dendritic Cells by B7-DC Cross-Linking Antibody Modulates T Cell Functions" was retracted in 2010. Reasons: an official misconduct investigation; misconduct by an author; results that could not be reproduced; concerns about the data.

### CD40 is necessary for IL-6 secretion by DC^XAb^ and reprogramming of Tregs to IL-17+ effectors

Treatment of DCs with B7-DC XAb leads to the production of IL-6 and IL-6-dependent conversion of T regulatory cells to IL-17+ effectors [5]. Blockade of NF-κB activation also prevents the secretion of cytokines including IL-6 from DC^XAb^ [6]. Thus, we sought to determine if these two responses of DC to B7-DC XAb were linked through a requirement for CD40. Wild type or CD40^−/−^ DCs were stimulated with control antibody or B7-DC XAb for 48 hours and the amount of IL-6 in the culture supernatants was determined by ELISA. Parallel cultures were stimulated with CD40 or TLR agonists. Wild type DCs secreted IL-6 when stimulated with B7-DC XAb or control stimuli targeting CD40 or toll-like receptors. Neither DC type secreted IL-6 when treated with control antibody. Importantly, CD40^−/−^ DCs did not secrete IL-6 when treated with anti-CD40 or B7-DC XAb antibodies, but were still able to respond to TLR stimulation (Fig. 3A).

**Figure 3:** DCs require CD40 in order to secrete IL-6 and convert Tregs to Th17 cells in vitro. (A) IL-6 was measured in culture supernatants of wild type or CD40^−/−^ (KO) DC stimulated for 48 h with control antibody, B7-DC XAb, anti-CD40 or TLR agonists as indicated. Statistical analysis was performed using one-way ANOVA. IL-6 secreted by WT DCs stimulated with B7-DC XAb was significantly higher than IL-6 secreted by WT DCs stimulated with control antibody; IL-6 secreted by wild type or CD40^−/−^ DC in response to TLR ligands was significantly higher than IL-6 induced in WT DC by B7-DC XAb (p<0.01). Error bars represent the standard deviation from the mean of triplicate cultures. (B) Enriched populations of DO11.10 non-Tregs or Tregs (>95% pure) were cultured with OVA-pulsed and control- or B7-DC XAb-treated DC isolated from wildtype, (C and E) CD40^−/−^ mice and (D) IL-6−/− mice. After 48 h, expression profiles for FoxP3 and IL-17A were determined by intracellular staining and flow cytometry. All experiments were conducted at least twice.

As a final test for the role of a CD40-NFκB-IL-6 pathway in the conversion of Tregs to T effector cells [5], wild type or CD40^−/−^ DC were pulsed with ovalbumin and treated with the control antibody or B7-DC XAb. These DCs were then used in vitro as stimulators of cultures enriched for either CD4^+^ CD25^+^ Tregs or CD4^+^ CD25^−^ non-Tregs isolated from DO11.10 TCR transgenic mice. After 48 hours, cells from each group were subjected to intracellular staining for the Treg specific transcription factor FoxP3 and the Th17 specific effector cytokine IL-17A. Non-Tregs that were stimulated with antigen-pulsed wildtype or CD40-deficient DC^cntrl^ or DC^XAb^ did not express FoxP3 or IL-17A (Fig. 3B). Tregs stimulated with antigen-pulsed wild type DC^XAb^ downregulated FoxP3 and expressed IL-17A. CD40^−/−^ DC^XAb^s did not mediate the conversion of T regulatory cells to IL-17+ effector cells (Fig. 3C) suggesting the necessity of IL-6 in this process. Wild type DC^cntrl^ and CD40^−/−^ DC^cntrl^ also failed to cause T regulatory conversion to T effector cells. However, it is possible that IL-6 alone is not sufficient for inducing DC^XAb^ mediated T regulatory cell conversion into effector cells. To test this, DC^cntrl^, DC^XAb^, CD40−/−^cntrl^, CD40−/−DC^XAb^, IL-6−/−^cntrl^ and IL-6−/−DC^XAb^ were analysed for their potential to induce T regulatory cell conversion by exogenous addition of IL-6. As shown in panels 3D and E, under culture conditions where the DCs are defective in making IL-6 (both IL-6−/− DCs and CD40−/−DCs), provision of IL-6 restored the induction of Th17 cells, whereas the CD40 deficient and IL-6 deficient DC^cntrl^ supplemented with IL-6 failed to induce IL-17A+ cells. This data indicate IL-6 is necessary, but not sufficient to cause T regulatory cell conversion to Th17 cells, highlighting the importance of other factors induced by B7-DC cross-linking in these regulatory events.

The article "Indirect Recruitment of a CD40 Signaling Pathway in Dendritic Cells by B7-DC Cross-Linking Antibody Modulates T Cell Functions" was retracted in 2010. Reasons: an official misconduct investigation; misconduct by an author; results that could not be reproduced; concerns about the data.

We have previously shown that DC^XAb^-mediated conversion of Tregs into IL-17+ effectors occurs in the absence of any significant cell proliferation [5]. Since the data in Fig. 3B show that non-Tregs did not express IL-17A after stimulation with DC^cntrl^ or DC^XAb^, we conclude that the IL-17A expressing cells originated from Tregs and were not a product of outgrowth of contaminating non-Tregs. These data show that CD40 is necessary for DCs to not only respond to B7-DC XAb by secreting IL-6, but also to induce the concomitant conversion of T regulatory cells into effector cells.

### CD40 is important for the generation of anti-tumor T cell responses induced by B7-DC XAb

A major response in mice receiving B7-DC XAb is the induction of a potent CTL response that drives the protection of those mice from a lethal melanoma challenge [18], [19]. To test the ability of the B7-DC XAb to confer protection against other tumor types, we injected cells derived from kidney, thymus, or breast tumors or leukemia or melanoma cells into genetically-matched hosts. Mice receiving each tumor type also received either control antibody or B7-DC XAb treatment. Nearly all of the mice (97%) that were treated with the control antibody succumbed to the tumor burden irrespective of the origin of the tumor or the tumor-host combination. Anti-tumor immunity was produced by B7-DC XAb treatment in either strain of mice tested and was also independent of tumor type (Table 1).

**Table 1:** B7-DC XAb Induces Protective Immunity Against a Variety of Different Tumor Grafts.

Tumor	Number of Cells	Mouse Strain	Number of Mice Tumor Free/Total (Control Ab)	Number of Mice Tumor Free/Total (B7-DC XAb)	p Value
B16	5×10^5^	C57BL/6	0/5	23/23	<0.001
RENCA	10^6^	C57BL/6	0/9	9/9	<0.001
EL4	5×10^5^	C57BL/6	0/8	8/8	<0.001
WEHI-3	5×10^3^	BALB/c	1/5	6/6	0.015
TUBO	5×10^5^	BALB/c	0/5	10/10	<0.001

Mice received B7-DC XAb or control antibody (i.v.) at the time they were grafted with tumor cells (s.c.). Mice were monitored regularly for tumor growth and were euthanized if tumors reached 17×17 mm. Mice remaining tumor-free were monitored regularly for up to 30 days; TUBO mice were monitored up to 300 days. The scores indicate the number of mice in the indicated treatment group remaining free of tumor.

The article "Indirect Recruitment of a CD40 Signaling Pathway in Dendritic Cells by B7-DC Cross-Linking Antibody Modulates T Cell Functions" was retracted in 2010. Reasons: an official misconduct investigation; misconduct by an author; results that could not be reproduced; concerns about the data.

CD40 has been shown to play a major role in cross-presentation of antigens to stimulate CD8 T cells [20], and anti-CD40 antibody treatment has been used to induce protection against tumors [10], [21]. Therefore, we analyzed the role of CD40 in the anti-tumor immunity elicited by B7-DC XAb in two tumor models. Wild type or CD40^−/−^ mice were implanted with B16 melanoma or WEHI-3 leukemia cells and treated systemically with the control antibody or B7-DCXAb. On day 7, lymph node cells were isolated from some of the treated mice and used as effectors against ^51^Cr-labeled B16 or WEHI-3 targets. EL-4 or P815 cells served as MHC-matched negative controls. In the CD40^−/−^ mice, potent effectors were not induced in response to B7-DC XAb treatment (Fig. 4). Moreover, when the remaining mice were followed for up to 90 days, we found that all the groups of mice succumbed to the tumor except the wild type mice receiving B7-DC XAb (Table 2). These data suggest that CD40 is necessary for the generation of the potent anti-tumor immunity induced by B7-DC XAb.

**Figure 4:** CD40 is required for the DC^XAb^-induced generation of anti-tumor CTL responses in vivo. Wild type or CD40^−/−^ mice were engrafted with B16 melanoma (A) or WEHI-3 leukemia (B) and treated intravenously with 30 µg B7-DC XAb or control antibody. On day 7, cells from draining lymph nodes were used as effectors in CTL assays. (A) CTL against ^51^Cr-labeled B16 tumor targets (Left) or unrelated EL-4 controls (Right). Filled squares show CTL for wild-type mice receiving B7-DC XAb. (B) CTL against ^51^Cr-labeled WEHI-3 tumor targets (Left) or unrelated, MHC-matched P815 controls (Right). Filled triangles show the CTL response from wild type mice receiving B7-DC XAb. Symbols and lines for all other treatment groups are nearly superimposable. The results shown are representative of 2 experiments.

**Table 2:** B7-DC XAb-induced Tumor Protection is Dependent on CD40.

Tumor	Mouse Strain	Number of Mice Tumor Free/Total (Control Ab)	Number of Mice Tumor Free/Total (B7-DC XAb)	p Value
B16	B6 WT	0/8	8/8	<0.001
B16	CD40−/−	0/8	0/8	n.s.
WEHI	BALB/cWT	0/3	5/5	<0.001
WEHI	CD40−/−	0/7	0/8	n.s.

Wild type or CD40−/− mice were implanted with B16 or WEHI tumor (5×10^5^ cells) and received control antibody or B7-DC XAb by intravenous administration. The mice were monitored for tumor growth and were euthanized if tumor size reached 17×17 mm. Tumor-free B16-implanted mice were monitored regularly for more than 90 days; tumor-free WEHI-implanted mice were monitored regularly for more than 60 days. The scores indicate the number of mice in the indicated treatment group remaining free of tumor. n.s. = not significant.

The article "Indirect Recruitment of a CD40 Signaling Pathway in Dendritic Cells by B7-DC Cross-Linking Antibody Modulates T Cell Functions" was retracted in 2010. Reasons: an official misconduct investigation; misconduct by an author; results that could not be reproduced; concerns about the data.

Since CD40 is expressed on multiple cell types, we asked whether the expression of CD40 on DC alone was critical for B7-DC XAb-induced anti-tumor immunity. To test this, bone marrow-derived wild type or CD40^−/−^ DCs were pulsed with B16 melanoma tumor cell lysate and treated with control antibody or B7-DC XAb. After overnight incubation, the DCs were adoptively transferred into normal mice as a vaccine. Mice were then implanted with live B16 tumor. The animals were followed for 90 days for the development of tumor. Whereas mice receiving wild-type DC^XAb^ vaccine were protected from melanoma challenge, animals receiving the CD40^−/−^ DC^XAb^ succumbed to the tumor (Table 3). Taken together, these data show that CD40 on DC is critical for B7-DC XAb to confer tumor immunity in vivo.

**Table 3:** DC^XAb^ Vaccination Requires CD40 for Tumor Immunity.

Tumor	Mouse Strain	Number of Mice Tumor Free/Total (Control Ab)	Number of Mice Tumor Free/Total (B7-DC XAb)	p Value
B16	WT	0/4	4/4	0.029
B16	CD40−/−	0/4	0/4	n.s.

Normal mice received 2×10^6^ wild-type or CD40^−/−^ DC pulsed with B16 tumor lysate and control antibody or B7-DC XAb as indicated. On the same day, 5×10^5^ B16 tumor cells were implanted on the right flank. The animals were monitored for tumor growth for at least 90 days and were euthanized if the tumor reached 17×17 mm. The scores indicate the number of mice in the indicated treatment group remaining free of tumor. n.s. = not significant.

## Discussion

Cross-linking dendritic cells with B7-DC XAb results in a number of phenotypic changes, including enhanced survival, increased ability to accumulate antigen, enhanced ability to activate naïve T cells, increased efficiency of seeding draining lymph nodes, and the up-regulation of key immunomodulatory cytokines [2], [22]–[24]. B7-DC has no known ability on its own to transduce an intra-cellular signal. Therefore, we have focused on delineating the events that occur on the surface of the DCs upon binding of B7-DC XAb and to determine what membrane and intracellular molecules mediate the various DC phenotypic responses. Previously, we found that cross-linking B7-DC induced a substantial reorganization of cell surface molecules, resulting in the clustering of MHC, CD80, CD86, and CD11c molecules into a cap [3]. In this report we document that CD40 is also present within this cell surface complex on DC^XAb^. The recruitment of CD40 is necessary for the B7-DC XAb-induced activation of NFκB and protection of DC from cell death signals, a response also linked to the secretion of cytokines such as IL-6. Moreover, CD40 expression is required for DC^XAb^-induced conversion of T regulatory cells to IL-17-producing effector cells in vitro and the induction of CTLs capable of conferring tumor-protective immunity in mice. However, under culture conditions where the DCs are compromised in their ability to secrete IL-6 in response to B7-DC XAb treatment, addition of exogenous IL-6 resulted in generation of IL-17 cells, albeit at a lesser frequency. Antigen presentation by DC^cntrl^ in the presence of exogenously added IL-6 fail to induce Treg conversion. This implies that apart from IL-6, other unknown factors from DCX^Ab^ are necessary to cause complete conversion of T regulatory cells. Taken within the context of our previous finding that TREM-2 recruitment on DC^XAb^ mediates the induction of antigen accumulation by mature DC [3], we conclude that B7-DC XAb has its many unique biologic effects due to its ability to specifically target the surface of DC, recruit, and activate common signaling pathways in DC that, in turn, modulate multiple T cell functions.

The article "Indirect Recruitment of a CD40 Signaling Pathway in Dendritic Cells by B7-DC Cross-Linking Antibody Modulates T Cell Functions" was retracted in 2010. Reasons: an official misconduct investigation; misconduct by an author; results that could not be reproduced; concerns about the data.

Dendritic cells treated with B7-DC XAb exhibit some similarities to DC activated by other means, but there are key differences. Typically, stimulation through TNFR, CD40, or TLR as well as through TREM-2 results in a maturation response in DC, which is associated with the up-regulation of CD80, CD86, and MHC class II and a decrease in antigen uptake [25], [26]. However, DC^XAb^ do not exhibit this classic “mature” phenotype. In fact, B7-DC XAb causes matured DC to regain the ability take up antigen [2], and it stimulates antigen presentation by immature DC [27]. B7-DC cross-linking has little effect on the levels of class II, CD80, and CD86, but upregulates CCR7 expression. CD40 ligation typically down-regulates TREM-2 [28], but our studies show that B7-DC XAb co-opts both CD40 and TREM-2 signals.

Many TLR and TNFR family members activate NFκB through MyD88 [29] whereas B7-DC XAb activation of NFκB is MyD88-independent [6]. Other cell surface receptors present on DC (TLRs, CD80, CD86, and TREM-1) can activate NFκB [29], but experiments with CD40^−/−^ DC suggest that CD40 is the one required by B7-DC XAb. TREM-2 binds DAP12 to activate Syk. Stimulation of DC via TREM-2 also induces a maturation response and activates ERK [25]. B7-DC XAb activates ERK, but ERK is not involved in the TREM-2 mediated response of DC to B7-DC XAb [3]. However, ERK activation was dependent on the expression of CD40 on the dendritic cells activated with B7-DCXAb. These findings suggest that the combined signals from CD40 and TREM-2 upon B7-DC cross-linking are different than when either signal is generated through traditional means, or that each of these signals (and perhaps other signals not yet delineated) are only partially “on” in DC^XAb^.

The article "Indirect Recruitment of a CD40 Signaling Pathway in Dendritic Cells by B7-DC Cross-Linking Antibody Modulates T Cell Functions" was retracted in 2010. Reasons: an official misconduct investigation; misconduct by an author; results that could not be reproduced; concerns about the data.

Thus, fundamental to the mechanism of action of B7-DC XAb is its ability to activate CD40 and TREM2 pathways in an indirect, but DC-specific manner. Cell-specific activation of multiple pathways is potentially advantageous from a therapeutic perspective, especially when it can be induced with a single reagent. Furthermore, B7-DC XAb is effective as a modulator of T cell functions in animal models, even in the absence of ex vivo manipulations. Teasing out additional details in the signals emanating from B7-DC XAb will be critical to furthering our understanding of how of this novel immune modulator works. For example, various TNF receptor associated factors (TRAFs) mediate a diverse array of events downstream of CD40 and related receptors [30]. A role for TRAFs in DC^XAb^ remains to be tested. Whether B7-DC XAb also activates other kinases that regulate NFκB (e.g., pim1 dependent kinase, [31]) is not known. Whether B7-DC XAb affects cIAP, Bcl molecules, or additional survival-promoting pathways is also not known.

The net effect of using this reagent in animal models is an antigen-specific modulation of immune responses resulting in the alleviation of allergic responses, the clearance of tumors, and the induction of specific autoimmunity [4], [5], [18], [19], [32]. Studies with B7-DC XAb have provided new insights into the plasticity of T cell lineages and have expanded the potential of immune-based therapies to impact disease. In this regard, we have shown that B7-DC XAb also activates human DC [6], allowing for results in mouse models to be rapidly translated into the clinic. Generation of such highly antigen specific immunity in the absence of autoimmunity with B7-DC XAb [5] suggests a hypothesis that IgM-based therapeutic antibodies provide a way to induce the integration of complex signals in a cell-specific manner. Testing of this hypothesis and translation of B7-DC XAb to treat human cancers is now underway.

## Materials and Methods

### Ethics Statement

All animals were handled in strict accordance with good animal practice as defined by the relevant national and/or local animal welfare bodies, and all animal work was approved by the Institutional Animal Care and Use Committee of Mayo Clinic (protocol numbers A10306, A207, and A33403).

### Mice and reagents

C57BL/6J mice, BALB/CJ mice, DO11.10 mice, CD40^−/−^ mice, and IL-6^−/−^ mice were purchased from The Jackson Laboratory (Bar Harbor, ME). Male mice were used, and all experiments were conducted with IACUC oversight. The B16 melanoma cell line was kindly provided by Dr. Richard Vile (Mayo Clinic, Rochester, MN) and the RENCA cell line was kindly provided by Dr. Eugene Kwon (Mayo Clinic, Rochester, MN). EL-4 and WEHI-3 lines were purchased from American Type Culture Collection (ATCC, Vanassas, VA). The TUBO cell line, derived from a spontaneous breast carcinoma in a Balb-neuT mouse [33], was a gift from Dr. Esteban Celis (Moffitt Cancer Center, Tampa, FL). All tumor cell lines were maintained in DMEM (Life Technologies Invitrogen) containing 10% cosmic calf serum (Hyclone). Anti-mouse CD4-PE (RM4-5), MHC class II specific IgM (25-9-3), and purified anti-mouse MHC class II(M5/114.15.2) were purchased from BD Biosciences (San Jose, CA). APC-coupled FoxP3 antibody (FJK-16s), anti-mouse IL-17A-PE (eBio17B7) and purified and PE-coupled anti-mouse CD40 (IC10) and APC-coupled anti-mouse MHC class II antibody (M5/114.15.2) were purchased from eBioscience (San Diego, CA). Antibody against Syk kinase (4D10) and ERK (C.14) was obtained from Santa Cruz Biotechnology (Santa Cruz, CA). Anti-phosphotyrosine (4G10), anti phospho ERK (9101) and Goat anti-mouse antibodies were obtained from Upstate Cell Signaling Solutions (Lake Placid, NY). Rabbit antibody against DAP12 (MC457) was developed by Dr. Paul Leibson (Mayo Clinic, Rochester, MN). Protein A-Sepharose was purchased from Pierce Biotechnology (Rockford, IL). For analysis of co-precipitating signaling molecules, affinity purified antibody against mouse Class II (I-A^b^) (KH74) (BD Biosciences, San Jose, CA) was used. Vitamin D_3_ (1α, 25-dihydroxyvitamin D_3_) was a gift from Dr. Matthew Griffin (Mayo Clinic, Rochester, MN). Receptor activator of the NF-κB (RANK) ligand was purchased from Chemicon International. The TLR ligands were used at 10 µg/ml and were as follows: TLR2 ligand, Pam3CSK4 (InVivogen); TLR3 ligand, polyI∶C (Calbiochem); TLR 4 ligand, LPS (Sigma); TLR7/8 ligand, Gardiquimod (InVivogen); TLR9 ligand, CpG (synthesized in Mayo core facility).

The article "Indirect Recruitment of a CD40 Signaling Pathway in Dendritic Cells by B7-DC Cross-Linking Antibody Modulates T Cell Functions" was retracted in 2010. Reasons: an official misconduct investigation; misconduct by an author; results that could not be reproduced; concerns about the data.

### B7-DC XAb

The human monoclonal IgM antibodies B7-DC XAb (sHIgM12) and isotype-matched control (sHIgM39) were identified in a screen for mouse DC-binding antibodies present in a bank of serum samples from patients with monoclonal gammopathies. The DC-binding sHIgM12 antibody and the non-binding sHIgM39 control antibody and were purified as described [1]. Because of the dependence on B7-DC for its biologic properties, the requirement for the pentameric form, and the observed signals in DC elicited by antibody binding, we refer to sHIgM12 as B7-DC cross-linking antibody (B7-DC XAb).

### Flow Cytometry and Fluorescence Resonance Energy Transfer (FRET)

Flow cytometry was used to quantify close molecular interactions on the cell surface as described previously [34]. Briefly, mouse DC were stained with anti-Class II-APC (M5/114.15.2) and anti-CD40-PE (IC10). All staining was for 15 minutes. Cells were stimulated with 10 µg/ml control antibody or B7-DC XAb or purified anti-mouse MHC class IIIgM (25-9-3) and aliquots from different groups were taken at different time points. The cells were washed and fixed in 2% paraformaldehyde prior to analysis by FACS performed by the Mayo Flow Cytometry Core Facility using a FACSCaliber (BD Biosciences, Franklin Lakes, NJ). FRET (upon excitation of PE at 488 nm and emission of APC at 660 nm) was visualized in FL3 channel (650–670 nm LP). Data collected as log_10_ fluorescence were analyzed using CellQuest (BD Biosciences). MFI = Mean Fluorescence Intensity.

### Isolation of Tregs and non-Tregs

Splenocytes were isolated from pooled spleens harvested from three mice. Tregs were isolated by positive selection using Mouse Treg Isolation kit from Miltenyi Biotec (Auburn, CA), as per the manufacturer's protocol [5]. Briefly, splenocytes were incubated with anti-CD25 antibody coupled to magnetic beads for 15 min prior to binding to the MACS column. Cells that were not bound were washed three times with RPMI/10% FBS and used as non-Tregs. Adherent cells (Tregs) were eluted and washed prior to use.

### In vitro activation of Tregs and non-Tregs

Bone marrow derived WT or CD40^−/−^ immature DCs (2×10^6^) were pulsed with antigen and treated with control antibody or B7-DC XAb overnight then used to stimulate naïve DO11.10 Tregs in culture (together in 24-well plates) at a 1∶1 ratio in vitro for 48 hours. After 48 hours, cells were removed, pooled, and prepared for analysis by intracellular staining for the expression of FoxP3 and IL-17A. In some experiments, 20 ng/ml of IL-6 (R&D Systems, Minneapolis) was added at the start of the culture. Briefly, cells were permeabilized with CytoFix/CytoPerm kit (BD Biosciences, San Diego, CA) and incubated with the appropriate conjugated antibody at 4°C according to the manufacturers' suggestions prior to analysis by flow cytometry as described [5].

### Generation of bone marrow DCs

DCs were generated from the mouse bone marrow [35]. Bone marrow cells were plated (1×10^6^/ml) in RPMI /10% serum containing 10 µg/ml of murine GM-CSF and 1 ng/ml of murine IL-4 (PeproTech, Rocky Hill, NJ). The culture medium was changed on day 2. DCs were used on day 6 unless otherwise indicated. For adoptive transfer experiments, day 6 DC were pulsed with antigen (1 mg/ml) and isotype control antibody or B7-DC XAb (10 µg/ml) overnight and injected into mice the following day.

The article "Indirect Recruitment of a CD40 Signaling Pathway in Dendritic Cells by B7-DC Cross-Linking Antibody Modulates T Cell Functions" was retracted in 2010. Reasons: an official misconduct investigation; misconduct by an author; results that could not be reproduced; concerns about the data.

### Confocal microscopy

Wild type or CD40^−/−^ DC were stimulated with 10 µg/ml of Ab or TLR ligand for 15 minutes, fixed and permeablized using Cytofix/Cytoperm kit (BD Pharmingen). Subsequently, Ab against a C-terminal peptide of NFκB was added followed by anti-rabbit FITC. Nuclei were stained with DAPI (Sigma-Aldrich) before being observed with a LSM510 laser scanning confocal microscope (Carl Zeiss) at 40× magnification and LSM510 software was used for the analysis.

### Cell viability assay

Wild type or CD40^−/−^ DCs were tested for their viability in a cytokine-deprived environment as previously described [6]. In brief, day 5 DCs were plated in triplicate into 96-well plates (2×10^4^ cells/well) in RPMI 1640 without serum, GM-CSF, or IL-4 and in presence of B7-DC XAb, isotype control Ab, or RANK ligand (10 µg/ml). For experiments using vitamin D_3_ to induce cell death [17], DCs were matured with 200 ng/ml CpG plus 10 nM vitamin D_3_. All cultures were maintained overnight then Alamar Blue (Biosource International) was added to a final concentration of 10% (v/v). Readings were taken after additional 24 h of culture using a Spectra Max M2 Multi Detection Reader (Molecular Devices) set to an excitation wavelength of 520 nm and an emission reading of 590 nm.

### Tumor experiments

All in vivo tumor experiments were carried out as previously described [19]. Briefly, mice (wild-type or CD40^−/−^) were injected with the indicated number of tumor cells in the right flank, and received control antibody or B7-DC XAb (30 µg) by intravenous administration. The mice were monitored regularly for tumor growth. To assess CTL responses, draining lymph node cells (from 2 mice in each group) were harvested on day 7, pooled, and used as effectors against the ^51^Cr-labeled B16 melanoma or WEHI-3 target and EL4 or P815 control cells. The remaining mice were monitored for tumor growth for the times indicated. For experiments using adoptive transfer of DC, mice received B16 melanoma lysate-pulsed wild type or CD40^−/−^ dendritic cells (2×10^6^, intraperitoneally) pretreated overnight with 10 µg/ml control antibody or B7-DC XAb. In all experiments, mice bearing tumors of size 17×17 mm were euthanized as per the Institutional Animal Care and Use Committee recommendations. Fisher exact probability test analyses were conducted using SigmaPlot software.

### IL-6 ELISA

Bone marrow-derived DC from wild type or CD40^−/−^ mice (1×10^6^ DC/well) were stimulated for 48 h with 10 µg/ml B7-DC XAb, control antibody, anti-CD40 antibody, or TLR ligand. Murine IL-6 was detected in culture supernatants using Ready-Set-Go ELISA kits from e-bioscience (San Diego, CA, USA) as per the manufacturer's instructions. Samples were run in triplicate and values are recorded as mean±standard error of the mean. Statistical analysis was performed by one-way ANOVA using Sigma Stat software.
